The article "Topological Organization Alterations of Whole-Brain Functional Networks in Patients with Childhood Absence Epilepsy: Associations with Treatment Effects" was published in 2021. Journal: Dis Markers.

# Topological Organization Alterations of Whole-Brain Functional Networks in Patients with Childhood Absence Epilepsy: Associations with Treatment Effects

**DOI:** 10.1155/2021/2727596

**Published:** 2021-06-26

**Authors:** Xueyu Wang, Peng Fang, Dongmei Jiao, Tian Hu, Qi Yang, Wei Liang, Yijun Li, Yibing Yan, Libo Liu

**Affiliations:** ^1^Department of Pediatrics, Shandong Provincial Hospital, Cheeloo College of Medicine, Shandong University, Jinan, Shandong 250021, China; ^2^Department of Pediatrics, Shandong Provincial Hospital Affiliated to Shandong First Medical University, Jinan, Shandong 250021, China; ^3^Department of Military Medical Psychology, Air Force Medical University, China; ^4^Department of Internal Medicine, The Second Affiliated Hospital of Shandong Traditional Chinese Medicine University, Jinan, China; ^5^Department of Radiology, Yanan University Affiliated Hospital, China; ^6^Department of Radiology, Affiliated Hospital of Shaanxi University of Traditional Chinese Medicine, China; ^7^Department of Pediatrics, The First Affiliated Hospital of Shandong First Medical University, Jinan, China; ^8^Department of Cardiology, The Second Affiliated Hospital of Shandong First Medical University, Taian, China

## Abstract

**Purpose:**

The purpose of the current study is to detect changes of topological organization of whole-brain functional networks and their relationship with the clinical treatment effects of antiepileptic drugs (AEDs) for patients with childhood absence epilepsy (CAE) using resting-state functional MRI (RS-fMRI). *Patients and Methods*. RS-fMRI data from 30 CAE patients were collected and compared with findings from 30 age- and gender-matched healthy controls (HCs). The patients were treated with first-line AEDs for 46.03 months before undergoing a second RS-fMRI scan.

**Results:**

CAE children at baseline showed a reduced clustering coefficient (Cp) and local efficiency (El) than the HC group, implying the reduction of functional segregation. CAE children at baseline also showed smaller characteristic path length (Lp) and higher global efficiency (Eg) compared with the HC group, implying the impairment of functional segregation. However, those metrics showed no significant differences between CAE children at follow-up and the HC group which indicated a clear renormalization of topological organization after AED treatments. CAE at follow-up also showed significantly decreased connectivity between several network regions, with which the thalamus is mainly involved. Furthermore, the reduced connectivity change between the left superior parietal gyrus and the left thalamus is positively correlated with the symptom improvements after AED treatment.

The article "Topological Organization Alterations of Whole-Brain Functional Networks in Patients with Childhood Absence Epilepsy: Associations with Treatment Effects" was published in 2021. Journal: Dis Markers.

**Conclusion:**

We highlighted the convergence and divergence of brain functional network dysfunctions in CAE patients and provided crucial insights into pathophysiological mechanisms and the AED effects.

## 1. Introduction

Childhood absence epilepsy (CAE) is the most common pediatric epilepsy syndrome, and its clinical features are transient (10-20 s) nonconvulsive seizures with impairment of consciousness [1]. Electrographically, absence seizures are characterized by a typical pattern of generalized 3 Hz spike and wave bursts with normal background activity [2]. Recently, noninvasive techniques of functional magnetic resonance imaging (fMRI) have played an important role in studying the neural mechanisms of epilepsy in the human brain [3]. Numerous efforts have been made to identify focal abnormalities of brain activity in CAE children, and higher-order association cortices (frontal cortex, parietal cortex) and subcortical (thalamus and putamen) and cerebellar regions are found to be the crucial regions in the initiation and propagation of absence seizure in patients with CAE [4]. However, CAE is thought of a dysconnectivity disorder in multiple connection circuits rather than a focal disturbance in a single brain area, and impairments of cortical-subcortical pathways have been identified [5]. As a powerful quantitative method for explaining the topological architecture of complex brain networks, graph-based connectivity analysis can reveal topological disorganization in the whole-brain network that can serve as markers for clinical diagnostic and also disease outcome estimation [6].

Medication is the primary and most commonly used treatment. The mainstay of treatment for epilepsy is antiepileptic drugs (AEDs). Ethosuximide (ETX), valproic acid (VPA), and lamotrigine (LTG) are commonly used to treat CAE [2]. However, few studies have evaluated longitudinal changes in brain activity after AED treatment. Investigations of brain changes before and after treatment can not only improve our understanding of the mechanisms and recovery of seizures but also help monitor treatment outcomes and guide the choice of the best treatment. Therefore, question raises that how the network architecture was influenced in children of CAE and whether the aberrant network organization could be adjusted along with clinical improvement after treatment.

Functional segregation and functional integration are two major fundamental organization principles of human brain functional network [7]. Functional segregation, which included clustering coefficient (Cp), normalized clustering coefficient (*γ*), and local efficiency (El), indicated specialized processing within interconnected brain regions, and functional integration, which included characteristic path length (Lp), normalized characteristic path length (*λ*), and global efficiency (Eg) indicated different brain areas in terms of functional and effective connectivity. The balance between segregation and integration is vital for effective information processing and synthesis. Another important principle of human functional network is small-worldness (*σ* = *γ*/*λ*), which is characterized by a high global integration and a high local specialization between brain regions. These characteristics enable the brain network to meet local and global demands and balance functional integration and segregation in order to achieve synchronization of neural activity between different brain regions. Some findings have been observed for temporal lobe epilepsy and epilepsy; however, few studies have studied the topological differences between CAE children and healthy controls and investigated the longitudinal network reorganization after AED treatment.

The article "Topological Organization Alterations of Whole-Brain Functional Networks in Patients with Childhood Absence Epilepsy: Associations with Treatment Effects" was published in 2021. Journal: Dis Markers.

To address these issues, the current study employed resting-state fMRI and graph theoretical approaches to investigate topological organization of whole-brain function networks in a group of CAE children who obtained resting-state fMRI data before and after AED treatment. We hypothesized that (1) CAE children would demonstrate reduced functional segregation and impaired network integration compared to healthy children. (2) These abnormal activities might reorganize after AED treatment, and (3) these network abnormalities would be associated with the clinical efficacy of AEDs.

## 2. Methods

### 2.1. Subjects

Thirty-five children (20 males) diagnosed as childhood absence epilepsy were recruited. Clinical diagnosis was based on the International League against Epilepsy (ILAE) classification and confirmed by EEG data. Subjects were excluded if they have other psychiatric, neurological diseases or any structural abnormalities detected by routine MRI examination. At 40-50 weeks after first fMRI recording, we performed follow-up assessments of all patients and gathered information about AEDs and prognosis. In addition, thirty age- and gender-matched healthy controls (HCs) were recruited by advertisement. The Shandong Provincial Hospital affiliated to Shandong First Medical University approved the present study. All participants and their guardians signed written informed consent forms.

### 2.2. Functional Magnetic Resonance Imaging Data Acquisition

GE 3.0 Tesla Discovery MR scanner with an eight-channel-phased array head coil (EXCITE, General Electric, Milwaukee, Wisconsin) was used to collect the imaging data. The subjects were asked to stay still and to stay awake during the entire session [3]. Using the gradient-echo planar imaging sequence, the resting-state functional images were obtained with the following parameters: repetition time = 2000 ms, echo time = 30 ms, field of view = 240 mm × 240 mm, data matrix = 64 × 64, slices = 33, and total 210 volumes. Using a volumetric three-dimensional spoiled gradient recall sequence, the high-resolution T1-weighted image was also acquired with the following parameters: repetition time = 8.2 ms, echo time = 3.2 ms, field of view = 256 × 256 mm [2], matrix = 128 × 128, slice thickness = 1 mm, and 196 slices in the axial plane. Same parameters were used for scans of follow-up assessment of CAE children and for healthy controls.

The article "Topological Organization Alterations of Whole-Brain Functional Networks in Patients with Childhood Absence Epilepsy: Associations with Treatment Effects" was published in 2021. Journal: Dis Markers.

### 2.3. fMRI Data Preprocessing

Preprocessing of fMRI data was conducted using the Data Processing and Analysis for Brain Imaging (DPABI) which synthesizes procedures in the Resting-State fMRI Data Analysis Toolkit (REST; http://www.restfmri.net) and Statistical Parametric Mapping (SPM12; http://www.fil.ion.ucl.ac.uk/spm) [8]. The first 10 images were removed to allow for magnetization equilibrium. The remaining 200 images were subjected to slice time correction, realigned motion (data were excluded if head motion exceeded 2 mm and 2°). Due to the heavy head motions, five CAE children were excluded for further analysis, and the final sample size includes 30 CAE children and 30 HCs. Individual T1-weighted images were coregistered to the mean of the realigned EPI images. The transformed T1 images were then segmented into gray matter, white matter, and cerebrospinal fluid. The diffeomorphic anatomical registration through exponentiated Lie algebra (DARTEL) tool was used to compute the transformation from individual space to MNI space and vice versa.

Resting-state fMRI measures were sensitive to microhead motions [9]. Therefore, the higher-level Friston-24 model (the 24 parameters include 6 head motion parameters, 6 head motion effects one time point before, and the 12 corresponding squared items) was regressed out of the realigned data. In addition, the mean frame-wise displacement (FD) was calculated as a measure of the microhead motion of each subject. Then, the nuisance signals were regressed out, including the average signals from the ventricles and white matter. We then spatially smoothed the images with a 6 mm full-width half-maximum isotropic Gaussian kernel. Finally, linear trends were removed from the time courses and temporal band-pass filtering was performed (0.01–0.08 Hz) [10].

### 2.4. Network Construction

GRETNA (http://www.nitrc.org/projects/gretna/) were used to analyze the network properties using graph theory [11]. Particularly, the automated anatomical labeling (AAL) atlas was used to parcellate the brain into 90 regions of interest (ROI). Pearson correlation coefficients between time series of all possible pairs of ROI were calculated, yielding a 90 × 90 correlation matrix for each participant. To ensure the number of nodes and connections were matched across participants, we used a sparsity threshold (8% ≤ *s* ≤ 50%) at the intervals of 0.01 to transform each correlation matrix into an undirected binarized matrix. Then, we computed the following measures: (1) the functional segregation metrics: clustering coefficient (Cp), normalized clustering coefficient (*γ*), and local efficiency (El); (2) functional integration metrics: characteristic path length (Lp), normalized characteristic path length (*λ*), and global efficiency (Eg); and (3) small-worldness metric: *σ* (*σ* = *γ*/*λ*). Similar with a previous study, we calculated the area under the curve (AUC) of for each network metric for further statistical comparisons [12]. Independent of single threshold selection, the AUC metric provides a summarized scalar for topological characterization of brain networks.

The article "Topological Organization Alterations of Whole-Brain Functional Networks in Patients with Childhood Absence Epilepsy: Associations with Treatment Effects" was published in 2021. Journal: Dis Markers.

### 2.5. Statistical Analysis

The chi-square test and Student's *t*-test were utilized to examine group differences in demographic characteristics and clinical data at baseline between patients and healthy controls with SPSS (IBM SPSS Statistics for Windows, version 18.0, IBM Corp.). For detection of between-group differences in global network measures, a two-sample *t*-test (healthy controls vs. patients from baseline; healthy controls vs. patients at follow-up) or paired *t*-test (baseline vs. follow-up) was used to identify the changes of AUC for each network metric. The threshold for significance was *p* < 0.05, corrected with the FDR criterion. The mean frame-wise displacement (FD) calculated during the preprocessing step was accounted by including this term as a covariate for each comparison. Finally, a network-based statistic (NBS) approach was used to determine any interregional connection that was significantly changed across the three groups [13].

Values of AUC for each network metric and each pairwise connectivity showing abnormal differences were extracted, and Pearson correlation coefficients were used to examine the associations between the changes in each network metric and clinical scores using SPSS. Correction for multiple comparisons was accomplished using the false discovery rate (FDR) method, with the “mafdr” script implemented in MATLAB [14].

## 3. Results

### 3.1. Demographic Information

All participants (CAE children and healthy controls) recruited in the current study are right-handed. The mean seizure frequency was 8.69 times each day, the mean age onset was 7.77 years, and the mean follow-up time was 46.03 weeks. The treatments for each CAE child are listed in Table 1. The mean FD values calculated during fMRI preprocessing showed no significant differences across the three groups (*p* = 0.70).

The article "Topological Organization Alterations of Whole-Brain Functional Networks in Patients with Childhood Absence Epilepsy: Associations with Treatment Effects" was published in 2021. Journal: Dis Markers.

### 3.2. Small-World Properties

Seven topologic small-world parameters were determined under a sparsity of 0.08 to 0.48 with an interval of 0.01. As shown in Figure 1, all the three groups had small-world properties (*λ* > 1, *γ* > 1, and *σ* > 1); however, no significant differences were found across the three groups. Significant differences were found for the functional segregation metrics Cp and El, and two-sample *t*-test indicated that CAE children at baseline showed reduced Cp (*t* = −4.29, *p* < 0.001) and El compared with HCs (*t* = −3.47, *p* < 0.001), whereas paired *t*-test indicated that CAE children at follow-up showed increased Cp (*t* > 5, *p* < 0.001) and El (*t* = 3.30, *p* < 0.001) compared with baseline; no significant differences were found between CAE children at follow-up and HCs, and results are shown in Figure 2. For functional integration metrics Lp and Eg, similar comparison results were found. CAE children at baseline showed decreased Lp compared with HCs (two-sample *t*-test, *t* = −3.19, *p* < 0.001) and follow-up (paired *t*-test, *t* = −3.19, *p* < 0.001); as for Eg, CAE children at baseline are higher than HCs (two-sample *t*-test, *t* = 4.01, *p* < 0.001) and follow-up (paired *t*-test, *t* > 5, *p* < 0.001), and results are shown in Figure 3.

### 3.3. Connectivity and Correlation Results

Compared to the baseline, CAE patients at follow-up showed decreased brain functional connectivity (Figures 4(a)–4(c)). These mainly occurred among the left olfactory (OLF), left amygdala (AMYG), right cuneus (CUN), bilateral fusiform (FFG), superior parietal gyrus (SPG), inferior parietal gyrus (IPL), right supramarginal gyrus (SMG), left putamen (PUT), bilateral pallidum (PAL), right superior temporal pole (TPOsup), bilateral middle temporal gyrus (MTG), right middle temporal pole (TPOmid), left medial superior frontal gyrus (SFGmed), and bilateral thalamus (THA). Those differences are statistically significant under NBS correction (*p* < 0.05). Furthermore, significant positive correlation was found between the change of epilepsy frequency and change of correlation coefficient between the left superior parietal gyrus and the left thalamus (Figure 4(d)).

## 4. Discussion

This study explores the abnormalities of brain network architecture and AED effect on CAE children using resting-state fMRI. At baseline, significantly reduced functional segregation and integration were found whereas these abnormalities showed a clear rebound at follow-up. Decreased region-region connectivity was also found, which is mainly involved the thalamus. Furthermore, the connectivity change between the left superior parietal gyrus and the left thalamus is positively correlated with the symptom improvements after AED treatment. Our results suggest that the involvement of specific regions in cortical and subcortical networks may be associated with the mechanisms of seizure generation and the neurological deficits observed in CAE patients and might shed new light about the AED effects on CAE patients.

The article "Topological Organization Alterations of Whole-Brain Functional Networks in Patients with Childhood Absence Epilepsy: Associations with Treatment Effects" was published in 2021. Journal: Dis Markers.

Numerous efforts have been made to identify focal abnormalities of the brain in CAE children. However, CAE is thought of as a dysconnectivity disorder in multiple neuronal circuits rather than a focal pathology in a single region [15]. Modeling the brain as a complex network in the context of graph theory will help to reveal topological disorganization in the whole-brain networks. Functional segregation and functional integration refer to the ability for local specialization and parallel information transfer in the brain network, respectively. One of the most significant characteristics of the healthy human brain network is a short path length and high transmission efficiency, known as small-world attributes. A balance between local segregation and global integration of signals associated with interconnected neurons allows efficient information transmission at low wiring cost and enables the brain network to meet local and global demands in order to achieve synchronization of neural activity between different brain regions. Both El and Cp are the metrics of functional segregation. The present study found that CAE children exhibited reduced local network efficiency (lower Cp and El), which indicate that the efficiency or “speed” of information transfer among the adjacent nodes, and the density of the local interconnectivity within a network is compromised. It might be plausible that the observed reduced local communication efficiency (functional segregation) of brain functional networks may arise from neurodevelopmental dysfunction such as excessive synaptic pruning in CAE children [16]. CAE patients also demonstrated abnormal enhanced functional integration (lower Lp and higher Eg) in the brain network. As functional integration ensures interregional prompt transfer of information in brain networks, the abnormal functional integration might lead to cognitive maldevelopment of higher-order cognitive tasks and conscious processing.

The significant connectivity changes in the thalamus are consistent with the known important role of the subcortical structure in the generalization of epileptic seizures [17]. The thalamus is involved in absence seizures as ictal activity during absence seizures has been found to propagate through cortico-thalamic-cortical pathways. The generation of absence seizures has been explained by a highly synchronized functional interplay between discrete thalamocortical regions [18]. Previous studies have found abnormalities of the thalamus in CAE patients including less GM volume [19], neuronal metabolic dysfunction, and white matter microstructural properties (fractional anisotropy) in the bilateral thalamus [20]. Long-term use of antiepileptic drugs may affect functional changes in CAE patients. A previous study reported similar results that significantly altered network organizations in the thalamus were found after surgery [21]. Another study that analyzed EEG characteristics in children with benign epilepsy reported significantly reduced discharges and significantly improved EEG findings after treatment [22]. As one core hubs in the brain network, the findings of the thalamus led us to conclude that these interventions may exert a therapeutic effect by engaging these disconnected hubs within the network architecture of the brain.

The article "Topological Organization Alterations of Whole-Brain Functional Networks in Patients with Childhood Absence Epilepsy: Associations with Treatment Effects" was published in 2021. Journal: Dis Markers.

The bilateral middle temporal gyrus, the right middle temporal pole, and the left medial superior frontal gyrus are the main regions of default mode network (DMN). The absence seizures in CAE mainly arise from regions of the brain that are associated with conscious awareness, and the DMN has been shown to be more significantly influenced than other resting-state networks. Using seed-based analysis and independent component analysis, previous studies have indicated the disruption of DMN in CAE [23, 24]. Consistent with these previous studies, the finding on the DMN core regions suggests that the graph theory-based evaluation of functional brain networks can provide detailed insight into the activity of a pathological brain and can also be regarded as a support for further treatment.

## 5. Conclusion

We showed a normalization of the brain network architecture in patients with childhood absence epilepsy after AED treatments, based on the findings of clear rebound of functional segregation, functional integration, and reduced connectivity within cortico-thalamic-cortical pathways. In addition, our results indicated the graph-theory-based analysis can serve as a sensitive measure to provide crucial insights into pathophysiological mechanisms of CAE.

## Figures and Tables

**Figure 1:** The typical small-world network architectures (*γ* > 1, *λ* ≈ 1, and *σ* > 1) across the sparsity. Blue lines represent the healthy controls, red lines represent the CAE children at baseline, and green lines represent CAE children at follow-up. No significant differences were found across the three groups.

The article "Topological Organization Alterations of Whole-Brain Functional Networks in Patients with Childhood Absence Epilepsy: Associations with Treatment Effects" was published in 2021. Journal: Dis Markers.

**Figure 2:** Functional segregation metrics Cp and El. The bar graph shows the value of significant AUC of the functional segregation parameters among the 3 groups. Black asterisks indicate significant differences (*p* < 0.001).

**Figure 3:** Functional integration metrics Lp and Eg. The bar graph shows the value of significant AUC of the functional segregation parameters among the 3 groups. Black asterisks indicate significant differences (*p* < 0.001).

**Figure 4:** (a–c) Reduced connectivity after AED treatment. (d) Correlation results between the connectivity change from the left superior parietal gyrus to the left thalamus and the symptom improvements after AED treatment.

**Table 1:** Demographics of the CAE patient.

Patients	Sex	Onset age	Seizure frequency	AEDs before MRI scan	Initial AEDs	AEDs added	Follow-up (weeks)
1	F	11	12	No	LTG	No	43
2	M	6	6	No	VPA	No	55
3	F	7	9	No	LTG	VPA	54
4	M	9	8	No	VPA	No	50
5	M	10	2	No	VPA	No	36
6	M	8	6	No	LTG	No	45
7	F	7	5	No	LTG	Lost	46
8	M	9	7	No	LTG	VPA	40
9	F	11	2	No	LTG	No	51
10	F	6	8	No	Lost	No	53
11	M	8	9	No	VPA	No	39
10	M	7	2	No	VPA	No	42
13	F	7	11	No	LTG	No	48
14	F	8	3	No	LTG	VPA	49
15	F	6	8	No	VPA	LTG	52
16	M	9	2	No	VPA	LTG	57
17	M	9	12	No	LTG	LEV	56
18	F	8	20	No	VPA	No	32
19	M	10	6	No	LTG	No	50
20	M	11	8	No	LTG	No	48
21	F	9	9	No	LTG	No	49
22	F	6	7	No	VPA	No	43
23	M	5	9	No	VPA	LTG	47
24	M	3	6	No	VPA	No	37
25	F	6	13	No	LTG	No	41
26	F	8	20	No	Lost	No	46
27	F	7	9	No	LTG	No	47
28	M	5	15	No	VPA	LTG	36
29	M	3	16	No	VPA	No	46
30	F	10	13	No	LTG	No	49

## Data Availability

The datasets generated during and/or analyzed during the current study are available from the corresponding author on reasonable request.
